# Central Composite Designed Fast Dissolving Tablets for Improved Solubility of the Loaded Drug Ondansetron Hydrochloride

This article has been retracted.

**DOI:** 10.1155/2022/2467574

**Published:** 2022-08-21

**Authors:** Chandrashekar Thalluri, Ruhul Amin, Jithendar Reddy Mandhadi, Amel Gacem, Talha Bin Emran, Biplab Kumar Dey, Arpita Roy, Mohammed S. Alqahtani, Moamen S. Refat, Sher Zaman Safi, Amnah Mohammed Alsuhaibani

**Affiliations:** ^1^Faculty of Pharmaceutical Science, Assam Down Town University, Panikhaiti, Guwahati, Assam 781026, India; ^2^Department of Physics, Faculty of Sciences, University 20 Août 1955, Skikda, Algeria; ^3^Department of Pharmacy, BGC Trust University Bangladesh, Chittagong 4381, Bangladesh; ^4^Department of Pharmacy, Faculty of Allied Health Sciences, Daffodil International University, Dhaka 1207, Bangladesh; ^5^Department of Biotechnology, School of Engineering & Technology, Sharda University, Greater Noida 201310, India; ^6^Radiological Sciences Department, College of Applied Medical Sciences, King Khalid University, Abha 61421, Saudi Arabia; ^7^Bioimaging Unit, Space Research Centre, Michael Atiyah Building, University of Leicester, Leicester LE1 7RH, UK; ^8^Research Center for Advanced Materials Science (RCAMS), King Khalid University, Postcode: 9004, Zip code: 61413, Abha, Saudi Arabia; ^9^Department of Chemistry, College of Science, Taif University, P.O. Box 11099, Taif 21944, Saudi Arabia; ^10^Faculty of Medicine, Bioscience and Nursing, MAHSA University, Jenjarom, 42610 Selangor, Malaysia; ^11^IRCBM, COMSATS University Islamabad, Lahore Campus, Lahore, Pakistan; ^12^Department of Physical Sport Science, College of Education, Princess Nourah bint Abdulrahman University, P.O. Box 84428, Riyadh 11671, Saudi Arabia

## Abstract

Ondansetron tablets that are directly compressed using crospovidone and croscarmellose as a synthetic super disintegrant are the subject of this investigation. A central composite, response surface, randomly quadratic, nonblock (version 13.0.9.0) 3^2^ factorial design is used to optimize the formulation (two-factor three-level). To make things even more complicated, nine different formulation batches (designated as F1–F9) were created. There were three levels of crospovidone and croscarmellose (+1, 0, -1). In addition to that, pre- and postcompressional parameters were evaluated, and all evaluated parameters were found to be within acceptable range. Among all postcompressional parameter dispersion and disintegration time, *in vitro* drug release experiments (to quantify the amount of medication released from the tablet) and their percentage prediction error were shown to have a significant influence on three dependent variables. Various pre- and postcompression characteristics of each active component were tested *in vitro*. Bulk density, tap density, angle of repose, Carr's index, and the Hausner ratio were all included in this analysis, as were many others. This tablet's hardness and friability were also assessed along with its dimension and weight variations. Additional stability studies may be conducted using the best batch of the product. For this study, we utilised the Design-Expert software to select the formulation F6, which had dispersion times of 17.67 ± 0.03 seconds, disintegration times of 120.12 ± 0.55 seconds, and percentage drug release measurements of 99.25 ± 0.36 within 30 minutes. Predicted values and experimental data had a strong correlation. Fast dissolving pills of ondansetron hydrochloride may be created by compressing the tablets directly.

## 1. Introduction

Super disintegrates are a novel class of agents created in recent years. Excipients such as “Super disintegrates” assist break apart compacted mass when used in a liquid environment. This is critical for products that need quick release [1]. These novel compounds have better disintegration efficiency and mechanical strength at lower concentrations. Super disintegrants are the basis for developing rapid dissolving pills (RDPs). Super disintegrants are important in dissolving and disintegrating pills. Choosing the right super disintegrant concentration is critical for fast disintegration and high dissolution rates [2]. The combination of swelling and water absorption by the formulation causes super disintegration. The swelling of super disintegrants increases the wetted surface of the carrier, boosting wettability and dispensability of the system [3–5]. The ideal super disintegrant concentration is determined by the disintegrant's critical concentration. When the super disintegrant concentration is below a certain level, the disintegration time of the tablet decreases, but when the concentration is higher, the disintegration time remains constant or even increases [6, 7]. Croscarmellose sodium (Vivasol, AcDiSol) is a starch-free cross-linked cellulose that expands 4-8 folds in 10 seconds via both swelling and wicking mechanisms. It also swells in two dimensions and is best adapted for direct compression or granulation. In contrast to croscarmellose sodium, crospovidone acts through capillary action. Get a water-insoluble, spongy tablet. It gives empirical models (linear and quadratic) that characterize the influence of processing factors on the response investigated. The experimental design technique reduced the number of trials, identified factor interactions, identified the ideal response within the experimental zone, and empirically modelled the data [8]. The experiments used a two-factor, three-level central composite design. This architecture explores quadratic response surfaces and allows for polynomial model building. Central composite design can estimate second and third order effects, discover interfactor interactions, and find response optimums [9].

In addition to treating nausea and vomiting caused by cancer treatment, ondansetron hydrochloride has been shown to have anxiolytic and neuroleptic characteristics. It is highly powerful, deliquescent and metabolized rapidly in the liver [10]. Because patients with nausea and vomiting cannot take oral anti emetics, 5-HT3 receptor antagonists like ondansetron hydrochloride were first created as injectable. This is because it is simpler to administer oral antiemetic medicines than intravenous. Noninjectable ondansetron hydrochloride fast-dissolving tablets are a superior choice for cancer patients suffering from nausea, vomiting, and swallowing difficulties. For oral or buccal absorption, it may increase bioavailability. In tablet format, ondansetron hydrochloride is a low-dose drug, therefore, diluent action is more pronounced [11]. For the optimization of a new quick dissolving tablet formulation, ondansetron hydrochloride was chosen as a medication candidate.

## 2. Materials and Methods

Gifts from Torrent Pharma in Ahmedabad, India, and the Wockhardt Research Centre in Aurangabad, India, included ondansetron hydrochloride, the crospovidone and croscarmellose sodium formulations, respectively. Mannitol directly compressible was made possible by the kind donations of Indian lactose spray dried from Strides Arco Labs in Bangalore, Glenmark Ltd. in Nashik, and Alkem Labs Pvt Ltd. in Mumbai (Pearlitol SD 200). Analytical reagent quality was found in all of the other substances.

### 2.1. Experimental Design

There is an embedded factorial or fractional factorial design in the core composite design, which is supplemented with a collection of star points to enable for curvature estimate. Each face of the factorial space has a star point in the face-centered central composite design [12]. The regression analysis of the statistically relevant variables was used to create the second-order regression models [13, 14]. Regression models are of the following type:

(1) $$\begin{array}{c} Y=B_{0}+B_{1}\;X_{1}+B_{2}X_{2}+B_{12}\;X_{1}\;X_{2}+B_{11}\;X_{12}+B_{22}\;X_{22}. \end{array}$$

Each factor-level combination of *X*1 and *X*2 is analyzed; *B*_*o*_ is an intercept; *B*_1_–*B*_22_ are regression coefficients. *Y* is the constructive response associated with each factor-level combination. Predicting dispersion time (*Y*1), disintegration time (*Y*2), and percentage drug release (*Y*3) from fast dissolving tablets was made possible via the application of polynomial equations derived from this optimization approach. The validity of the response surface models was further evaluated by comparing predicted values for *Y*1, *Y*2, and *Y*3 with experimental data.

### 2.2. UV Absorption Spectroscopy

Using UV spectroscopy, it was determined that the drug concentration had been discovered. For the stock solution, the ondansetron hydrochloride was dissolved in a pH 6.8 phosphate buffer. A volumetric flask of 100 mL was used to transfer 100 mg of medicine. Using pH 6.8 phosphate buffer, the volume of stock solution (B) was brought up to the mark by diluting one mL of stock solution A with 100 mL of the buffer. For this experiment, aliquots of stock solution (B) (pH 6.8 phosphate buffer) were serially diluted from 2 to 20 microgram of drug per millilitre (mcg/mL). The absorbance of the final solutions was measured at 248 nm using a Systronics AU-2701 spectrophotometer in Mumbai, India [15].

### 2.3. Fourier Transform Infrared Spectroscopy (FTIR)

The FTIR spectra of the pure drug and the drug combination with super disintegrants were both reported. FTIR spectroscopy was used to evaluate the materials using the KBr pellet technique [7]. An equal amount of dry potassium bromide and 10 milligrams of the formulation are then blended together. Pestle and mortar are used to grind the mixture to a fine powder. A hydraulic press compresses the mixture into pellets. The findings were obvious when the transparent pellets were scanned using a frequency range of 4000–400 cm-1 [16].

### 2.4. Preparation of Ondansetron Hydrochloride Fast Dissolving Tablets by Direct Compression

By using the direct compression approach, it was possible to create ondansetron pills that dissolve quickly. Step by step, each component was combined, then sieved (number 100), and mixed with the medicine in a plastic bag for 15 minutes. At the end of this powder combination, talc and magnesium stearate were added and stirred for another 5 minutes. A single punch tablet machine was used to compress the active mixes into 200 milligram tablets. Preliminary batch findings were used to create 3^2^ factorial designs with two independent variables, *X*_1_ and *X*_2_, where *X*_1_ represents the quantity of crospovidone, and *X*_2_ represents the amount of croscarmellose in the final formulation. For each component, three levels (-1, 0, and +1) were chosen to represent low, centre, and high values [17]. There were at least nine batches of fast-dissolving tablet formulations evaluated before and after compression. Tables 1 and 2 show the arrangement and content of 3^2^ factorial designs for the ondansetron fast dissolving tablet formulation [18].

Where +1 is the high value, −1 is the low value, and 0 is the centre value for the factors *X*_1_ and *X*_2_. *X*_1_ is the amount of crospovidone, *X*_2_ is the amount of croscarmellose.

### 2.5. Precompression Parameters

Analysis of the precompression properties of each batch was carried out in accordance with established protocols, such as angle of repose, bulk density, tapped density, the Carr's consolidation index, and the Hausner's ratio [19].

### 2.6. Evaluation Parameters

#### 2.6.1. Weight Variation Test

Each of the 20 pills was weighed separately using a computerized weighted scale (Ohaus, USA). Calculate the average weight of 20 pills and compare the individual tablet weights (Table 3) [20, 21].

#### 2.6.2. Thickness

Placing the tablet between two arms of the vernier calliper (Indian calliper industries, Ambala, India), three pills from each batch were tested for thickness [20].

#### 2.6.3. Hardness

Tablet tensile strength (kg/cm^2^) is the force required to compress a tablet. The Monsanto Hardness Tester was used here (Perfit). A random selection of three tablets from each batch was made [22].

#### 2.6.4. Friability Test

Friability was assessed using a Roche friabilator. Twenty pills from each formulation were weighed and spun for four minutes at a speed of 25 resolution per minute. Removed any excess powder and then counted. The formula for determining how much weight one has lost is

(2) $$\begin{array}{c} \%Friability=W_{1}-W_{2}\times \frac{\;100}{W_{1}}. \end{array}$$

*W*_1_ is the pretest weight, and *W*_2_ is the posttest weight.

#### 2.6.5. Dispersion Time

Five 10 cm diameter tissue sheets were put in a petri plate (10 cm diameter). 10 mL eosin-water soluble dye was put to petri plate. On the tissue paper was carefully put a tablet. Wetting time is the time it takes for water to reach the tablet's top surface [22].

### 2.7. In Vitro Disintegration Test

For this test, the USP disintegration device was employed. Tested in 900 mL water at 37°C with six pills per formulation, the study was tripled [22].

### 2.8. In Vitro Drug Release Studies

The dissolving device USP II was used for this. At 37°C and 50 rpm, 900 mL pH 6.8 phosphate buffers were used for *in vitro* dissolving experiments. Five-minute aliquots were taken and analyzed at 248 nm on an Indian Systronics AU-2701 in Mumbai, India, at intervals of 5, 10, 15, 20, 25, and 30 minutes each. This was followed by a gradual release of medicines. There were three blindfolds in the test [23].

### 2.9. Accelerated Stability Studies

For three months, the stability of selected tablet batches was investigated in a stability chamber at 40°C and 75% RH (Remi Instruments, India). To determine the stability of a tablet formulation, the physical characteristics of the tablet were measured at various temperatures and times. It was determined that *in vitro* dissolving time and dispersion time were evaluated after 15 days, one month, two months, and three months.

## 3. Results and Discussion

### 3.1. FTIR Spectroscopy

Figures 1 and 2 show IR spectra of pure drug (ondansetron hydrochloride) and optimized formulation F6 drug with super disintegrates (crospovidone and croscarmellose). Ondansetron hydrochloride has large IR absorption peaks at 3941.01 and 3892.17 perhaps owing to OH hydrogen bonding. Carbonyl group vibrations at 1754.8 and 1684.67 may be responsible for peak 2983.77, including 1754.78. Ring stretching may be seen in 1556.22, 1508.11, and 1507.27, and the existence of all drug peaks in the IR spectrum of the drug polymer combination shows no drug-carrier interaction.

### 3.2. Precompression Parameters

Table 4 shows the precompression results of final active blends (F1–F9). Bulk and tapped densities varied from 0.571 ± 0.01 to 0.584 ± 0.02 and 0.610 ± 0.02 to 0.627 ± 0.060, respectively. Carr's index (12.14 ± 0.18 to 17.12 ± 0.21) and Hausner's ratio (1.14 ± 0.13 to 1.24 ± 0.17) data also revealed favorable flow qualities.

### 3.3. Postcompression Parameters

Table 3 shows the outcomes of postcompression investigations. All nine formulations were similar in size and hardness, ranging from 3.25 ± 0.14 to 3.41 ± 0.03. The low friability (1%) suggested good abrasion resistance. They passed the weight fluctuation test. All formulations had disintegration times under three minutes. The formulation that comprises F1, F3, and F6 formulations showed 37.13 ± 0.03 to 17.67 ± 0.03 and 147.25 ± 0.24 to 120.12 ± 0.55. However, the disintegration qualities are not preferred when the quantity of both super disintegrants is arbitrarily changed from high to low. The dispersion time for F4 and F8 formulations ranged from 130.25 ± 0.28 to 135.42 ± 0.29. Following the aforesaid observation, combining both disintegrates (7.5 percent of the total weight of tablet) has demonstrated a substantial effect and retards the optimal dispersion and disintegration time. The formulation of F6 revealed decrease dispersion and disintegration time of 17.67 ± 0.03 and 120.12 ± 0.55, respectively. So, the optimal doses of both super disintegrants were added to improve the dissolving properties of formulation F6 (99.25 ± 0.03). Based on disintegration and dissolving statistics, this formulation seems promising.

### 3.4. In Vitro Drug Release Studies

Figure 3 shows the *in vitro* drug release of each final formulation batch (F1–F9). In all batches, more than 80% of the medication was released within 30 minutes. Increased super disintegrant concentration increases drug release considerably, as in the F6 formulation. More F1–F3–F6 batches were soluble due to myriad disintegration mechanism established by the combination of both super disintegrants than F7–F9. The most critical stage is caused by the swelling impact of additional water penetration. When disintegration comes into touch with an appropriate medium, it swells. Thus, the adhesion force between the tablet's ingredients is overcome, resulting in the tablet disintegrating. The dissolving results indicated that the F6 formulation was the most promising batch, because the amount of drug release was found to be 99.25 ± 0.03 in 30 minutes.

### 3.5. Factorial Design

#### 3.5.1. *In Vitro* Disintegration Time

Crospovidone and croscarmellose concentrations were shown to affect disintegration time using a response surface plot (DT). According to the above findings, the disintegration times obtained were 147.25 ± 0.24 to 120.12 ± 0.55 seconds, with the polynomial equation producing a negative effect on disintegration time as concentrations of super disintegrates increased. This meant that as concentrations of super disintegrates increase, the disintegration time decreased. F4 and F8 were also found to have disintegration times of 130.25 ± 0.28 and 135.42 ± 0.29 seconds, respectively, based on the high-to-low-level or low-to-high-level disintegration levels. The capillary action of crospovidone super disintegrate has a more negative impact than that of croscarmellose, based on this finding. A random variation in disintegration time was seen because the concentrations of disintegrants could be varied from low to high levels, and the disintegration time was reduced from 142.21 ± 0.09 to 123.14 ± 0.17 seconds in this study.

Here is a model equation that can explain the disintegration time of a parameter.

(3) $$\begin{array}{c} Disintegration\;time=+133.42-9.05\;X_{1}-6.51\;X_{2}. \end{array}$$

Coefficient values in the polynomial equation were discovered to be negative in proportion to the decay continuance of each super disintegrant as a result of increasing super disintegrant concentrations. The results are shown in Figures 4 and 5, respectively.

#### 3.5.2. Dispersion Time

Crospovidone and croscarmellose were shown to affect dispersion time via the use of a response surface plot [24, 25]. Based on these findings, it can be concluded that the dispersion times obtained for crospovidone and croscarmellose are in the range of 37.13 ± 0.03 to 17.67 ± 0.03 seconds, with the polynomial equation producing a negative effect on dispersion time. This means that as concentrations of super disintegrates rise, so does the time required for their decomposition to take place.

As an additional measure, the dispersion time response was tested using two formulations: F4 which had high levels of crospovidone while having low levels of croscarmellose, and F8 which contained low levels while having a high level of crospovidone. After calculating the polynomial equation for both formulations F4 and F8, we found that the dispersion time was 22.24 ± 0.05 seconds for F4 and 27.74 ± 0.04 seconds for F8 when the concentration of each disintegrates or independent variable changed significantly. If you have ever had to break a pill in half because of a lack of super disintegrant, you will know what I am talking about.

Although the dispersion time of formulations including F2, F5, F7, and F9 was arbitrarily adjusted due to the concentrations of disintegrates being able to be modified from low to high, the disintegration time eventually decreased to be 33.48 ± 0.01 to 19.83 ± 0.01 seconds. Using the following model equation, dispersion time may be explained.

(4) $$\begin{array}{c} Dispersion\;time=+25.50-6.44\times X_{1}–3.48\times X_{2}+1.21\times X_{1}\times X_{2}+1.15\;X_{1}^{2}–0.4550\times X^{2}. \end{array}$$

The coefficient values of the polynomial equation were found to have a negative effect on wetting time when the concentrations of both disintegrates were at their highest, and a positive coefficient effect was found when the concentrations of the super disintegrate fluctuated randomly between the highest and lowest levels [26, 27]. Figures 6 and 7 depict the findings.

### 3.6. Percentage Drug Release

The dispersion time was shown to be affected by the quantity of crospovidone and croscarmellose in the solution [28]. The percentage drug release (percent) was found to range from 90.25 ± 0.41 to 99.25 ± 0.36 within 30 minutes, and the polynomial equation producing the positive effect on percentage drug release indicates that, as the concentration of super disintegrates increase, the percentage drug release increases [27, 29].

For this reason, the formulations F4 and F8, which contain low levels of crospovidone but high concentrations of croscarmellose, respectively, were created to guarantee that the interaction between two independent variables may affect drug release percentages in a positive manner. According to the polynomial equation, the change in concentration of either disintegrates or the independent variable displayed on the dependent response variable, i.e., the percentage drug release, was determined to be 94.78 ± 0.31 and 92.78 ± 0.15 within 30 minutes for formulations F4 and F8, respectively. A random variation in disintegration time was observed because the concentrations of disintegrates could be changed from low to high level, and thus, the percentage drug release was found to be between 91.18 ± 0.39 and 97.13 ± 0.23 within 30 minutes, despite the fact that the formulations contained F2, F5, and F7 as well. Figure 3 depicts the findings: as a result, the model equation for percentage medication release may be summarized as follows:

(5) $$\begin{array}{c} Percentage\;drug\;release\;\left(30\;minutes\right)=+94.17+2.82\;X_{1}+1.50\;X_{2}. \end{array}$$

Regression and ANOVA summaries, as well as a three-dimensional RSM plot for drug release percentage, are provided in Tables 5 and 6, respectively. Dispersion time, disintegration time, and *in vitro* drug release are all shown in Figures 8 and 9 by 2D and 3D RSM plots.

### 3.7. Numerical Optimization

Figure 10 demonstrates the numerical optimization process used to produce a new formulation with desired answers. Crospovidone and croscarmellose concentration combinations with a desire of 0.9705 met the highest criteria of an optimal formulation during the study. Various dependent variables were tested with the improved formulation. Data was gathered and analyzed to see whether the observed results matched those expected (regression values such as adjusted *R*^2^ and predicted *R*^2^ values). Results are shown in Tables 6 and 7 along with percent prediction errors for actual and projected responses.

### 3.8. Accelerated Stability Studies

For 90 days, stability investigations were conducted under accelerated stability conditions (40°C/75 percent RH) using an optimal batch F6 according to ICH recommendations. Formulation F6 (physical-chemical characteristics and release profile) showed no notable modifications, as reported in Table 8. There is a high degree of stability in the formulation even when subjected to extreme stress. As shown in Figure 3, the *in vitro* drug release curves for the F6 tablet after three months of stability testing are parallel to those of the initial F6 batch (prior to stability). This shows there has been no change in the drug release behavior of the F6 tablet after three months of stability testing. In addition to that, optimized formulation F6 ondansetron hydrochloride was compared to that of marketed formulation (Zofran ODT), and the results were noticed and concluded that their significant changes were recorded by comparing the percentage drug release within 30 minutes.

## 4. Conclusion

Ondansetron hydrochloride fast-dissolving tablets were developed and improved utilizing a central composite, response surface, randomized, quadratic, nonblock (13.0.9.0 version) 3^2^ factorial design. On the basis of early research, two independent variables, crospovidone and croscarmellose, were chosen. There were three levels of each of these independent variables. Dispersion time, disintegration properties, and drug release are all significantly affected by the abovementioned combination of super disintegrants, such as crospovidone and croscarmellose, at the same proportion (7.5% with formulation F6). Due to water penetration, the tablet's adhesiveness is overcome, causing the tablet to dissolve and break apart. Fast dissolving tablets' maximum release of medication was made possible by the combination of tablet porousness and disintegrate wicking characteristics. Optimum formulas were selected via feasibility and grid searches using Design-Expert software to optimize and construct response surface plots and contour plots. Multivariate regression analysis yielded statistically meaningful polynomial mathematical models for a variety of response variables. The Design-Expert programmed picked formulation F6 because it had a dispersion time of 17.67 ± 0.03 seconds, a disintegration time of 120.12 ± 0.55 seconds, and an *in vitro* drug release of 99.25 ± 0.36 percent within 30 minutes.

## Figures and Tables

**Figure 1:** FTIR spectra of pure drug (ondansetron hydrochloride).

**Figure 2:** FTIR spectra of optimized formulation F6 ondansetron hydrochloride fast dissolving tablets.

**Figure 3:** Cumulative percentage drug release of ondansetron hydrochloride fast dissolving tablets.

**Figure 4:** 2D contour plot graph for disintegration time with crospovidone and croscarmellose.

**Figure 5:** 3D RSM plot graph for disintegration time with crospovidone and croscarmellose.

**Figure 6:** 2D contour plot graph for dispersion time with crospovidone and croscarmellose.

**Figure 7:** 3D RSM plot graph for dispersion time with crospovidone and croscarmellose.

**Figure 8:** Contour plot graph for percentage drug release with crospovidone and croscarmellose.

**Figure 9:** 3D RSM plot graph for percentage drug release with crospovidone and croscarmellose.

**Figure 10:** Overlay plot graph of ondansetron fast dissolving tablets.

**Table 1:** Variables in 3^2^ full factorial design.

Formulation code	*X*_1_	*X*_2_
F1	0	0
F2	+1	0
F3	-1	-1
F4	+1	-1
F5	0	-1
F6	+1	+1
F7	-1	0
F8	-1	+1
F9	0	+1

**Table 2:** Composition of 3^2^ factorial design formulations of ondansetron hydrochloride fast dissolving tablets.

Name of ingredients in mg	F1	F2	F3	F4	F5	F6	F7	F8	F9
Ondansetron hydrochloride	10	10	10	10	10	10	10	10	10
Crospovidone (%*w*/*w*)	0	7.5	2.5	7.5	5	7.5	2.5	2.5	0
Croscarmellose (%*w*/*w*)	0	5	2.5	2.5	2.5	7.5	5	7.5	7.5
Spray dried lactose	150	150	150	150	150	150	150	150	150
Mannitol	q.s.	q.s.	q.s.	q.s.	q.s.	q.s.	q.s.	q.s.	q.s.
Magnesium stearate	7.5	7.5	7.5	7.5	7.5	7.5	7.5	7.5	7.5
Talc	7.5	7.5	7.5	7.5	7.5	7.5	7.5	7.5	7.5

**Table 3:** Evaluation of postcompressional parameters of factorial design formulations of ondansetron fast dissolving tablets.

Parameters	F1	F2	F3	F4	F5	F6	F7	F8	F9
Hardness (kg/cm^2^)	3.41 ± 0.03	3.25 ± 0.14	3.34 ± 0.02	3.42 ± 0.40	3.37 ± 0.41	3.27 ± 0.19	3.38 ± 0.02	3.31 ± 0.04	3.34 ± 0.09
Friability (%)	0.54 ± 0.04	0.54 ± 0.02	0.560 ± 0.02	0.52 ± 0.09	0.58 ± 0.08	0.54 ± 0.02	0.57 ± 0.05	0.56 ± 0.01	0.60 ± 0.04
Weight variation test (mg)	201.12 ± 0.17	200.15 ± 0.19	201.24 ± 0.32	198.15 ± 0.74	200.14 ± 0.23	200.21 ± 0.25	200.01 ± 0.17	200.25 ± 0.18	202.38 ± 0.19
Dispersion time (seconds)	25.49 ± 0.02	19.83 ± 0.01	37.13 ± 0.03	22.24 ± 0.05	28.50 ± 0.04	17.67 ± 0.03	33.48 ± 0.01	27.74 ± 0.04	21.59 ± 0.02
Disintegration time (seconds)	132.13 ± 0.15	123.14 ± 0.17	147.25 ± 0.24	130.25 ± 0.28	142.21 ± 0.09	120.12 ± 0.55	145.12 ± 0.12	135.42 ± 0.29	125.14 ± 0.28
Percentage drug release (%)	93.87 ± 0.12	97.13 ± 0.23	90.25 ± 0.41	94.78 ± 0.31	93.14 ± 0.25	99.25 ± 0.36	91.18 ± 0.39	92.78 ± 0.15	95.12 ± 0.14

Data are represented as mean ± SD (*n* = 3).

**Table 4:** Evaluation of precompression parameters of factorial design formulations of ondansetron hydrochloride fast dissolving tablets.

Parameters	F1	F2	F3	F4	F5	F6	F7	F8	F9
Bulk density (g/mL)	0.582 ± 0.01	0.584 ± 0.02	0.576 ± 0.01	0.572 ± 0.04	0.573 ± 0.02	0.571 ± 0.01	0.572 ± 0.01	0.574 ± 0.01	0.573 ± 0.02
Tapped density (g/mL)	0.614 ± 0.01	0.612 ± 0.02	0.610 ± 0.02	0.621 ± 0.08	0.618 ± 0.01	0.614 ± 0.02	0.622 ± 0.04	0.627 ± 0.06	0.615 ± 0.03
Angle of repose	21.14 ± 0.13	25.24 ± 0.31	22.34 ± 0.21	23.17 ± 0.21	22.21 ± 0.06	25.30 ± 0.51	24.72 ± 0.21	25.17 ± 0.08	25.48 ± 0.52
Carr's index	17.12 ± 0.21	12.27 ± 0.17	15.17 ± 0.11	13.54 ± 0.25	12.14 ± 0.18	15.02 ± 0.19	15.22 ± 0.21	14.12 ± 0.41	15.90 ± 0.25
Hausner ratio	1.22 ± 0.11	1.14 ± 0.13	1.24 ± 0.17	1.17 ± 0.21	1.15 ± 0.24	1.18 ± 0.22	1.19 ± 0.27	1.16 ± 0.15	1.14 ± 0.14

Data are represented as mean ± SD (*n* = 3).

**Table 5:** Response parameters of various formulations.

Formulation code	Concentration of CP (*X*1)	Concentration of CCM (*X*2)	Dispersion time in seconds	Disintegration time in second	Percentage drug release (%)
F1	5	5	25.49 ± 0.02	132.13 ± 0.15	93.87 ± 0.12
F2	7.5	5	19.83 ± 0.01	123.14 ± 0.17	97.13 ± 0.23
F3	2.5	2.5	37.13 ± 0.03	147.25 ± 0.24	90.25 ± 0.41
F4	7.5	2.5	22.24 ± 0.05	130.25 ± 0.28	94.78 ± 0.31
F5	5	2.5	28.50 ± 0.04	142.21 ± 0.09	93.14 ± 0.25
F6	7.5	7.5	17.67 ± 0.03	120.12 ± 0.55	99.25 ± 0.36
F7	2.5	5	33.48 ± 0.01	145.12 ± 0.12	91.18 ± 0.39
F8	2.5	7.5	27.74 ± 0.04	135.42 ± 0.29	92.78 ± 0.15
F9	5	7.5	21.59 ± 0.02	125.14 ± 0.28	95.12 ± 0.14

Data are represented as mean ± SD (*n* = 3).

**Table 6:** Summary of results of regression analysis and ANOVA for measured response.

Parameters	Response	*B*_*o*_	*B*_1_	*B*_2_	*B*_12_	*B*_11_	*B*_22_	Model lack of fit
Dispersion time in seconds	Coefficients	25.49	-6.43	-3.47	1.20	1.15	-0.45	Insignificant
	*P* value	—	0.0001	0.0002	0.0086	0.0249	0.1982	
	Regression	DF = 5	MS = 65.99	SS = 329.94	*F* = 432.20	*R* ^2^ = 0.9986	—	

Disintegration time seconds	Coefficients	133.42	-9.05	-6.51	—	—	—	Insignificant
	*P* value	—	<0.0001	0.0003	—	—	—	
	Regression	DF = 2	MS = 372.47	SS = 744.94	*F* = 81.80	*R* ^2^ = 0.9646	—	

Percentage drug release	Coefficients	94.17	2.82	1.50	—	—	—	Insignificant
	*P* value	—	<0.0001	0.0006	—	—	—	
	Regression	DF = 2	MS = 30.66	SS = 61.32	*F* = 96.41	*R* ^2^ = 0.9698	—	

**Table 7:** Comparison of regression values (*R*^2^) with the prediction error.

Response parameters	Constraints set	*R* ^2^ values	Adjusted *R*^2^ values	Predicted *R*^2^ values	% prediction error	Suggested model	*P* values
Dispersion time	Minimize	0.9986	0.9963	0.9831	0.518	Quadratic model	0.0465
Disintegration time	Minimize	0.9646	09528	0.9186	2.554	Linear model	<0.0001
*In vitro* drug release	Maximize	0.9698	0.9598	0.9167	0.675	Linear model	<0.0001

**Table 8:** Stability studies of optimized batch F6 at accelerated condition.

Time	Tablet thickness	Tablet diameter	Hardness (kg/cm^2^)	Friability (%)	Dispersion time (seconds)	Disintegration time (seconds)	Percentage drug release (%)
15 days	3.36 ± 0.04	8.02 ± 0.01	3.27 ± 0.19	0.54 ± 0.02	17.67 ± 0.03	120.12 ± 0.55	99.25 ± 0.36
30 days	3.38 ± 0.04	8.04 ± 0.01	3.20 ± 0.21	0.52 ± 0.01	19.14 ± 0.07	123.21 ± 0.36	98.34 ± 0.17
60 days	3.41 ± 0.03	8.11 ± 0.03	3.24 ± 0.14	0.53 ± 0.01	18.35 ± 0.04	125.31 ± 0.18	97.35 ± 0.28
90 days	3.43 ± 0.04	8.13 ± 0.05	3.21 ± 0.16	0.53 ± 0.04	17.54 ± 0.04	124.12 ± 0.39	96.28 ± 0.41

Data are represented as mean ± SD (*n* = 3).

## Data Availability

The data used to support the findings of this study are included within the article.
